# Advances regarding Neuroinflammation Biomarkers with Noninvasive Techniques in Epilepsy

**DOI:** 10.1155/2021/7946252

**Published:** 2021-12-22

**Authors:** Hongrui Ma, Hua Lin

**Affiliations:** Department of Neurology, Xuanwu Hospital, Capital Medical University, Beijing, China 100053

## Abstract

A rapidly growing body of evidence supports that neuroinflammation plays a major role in epileptogenesis and disease progression. The capacity to identify pathological neuroinflammation in individuals with epilepsy is a crucial step on the timing of anti-inflammatory intervention and patient selection, which will be challenging aspects in future clinical studies. The discovery of noninvasive biomarkers that are accessible in the blood or molecular neuroimaging would facilitate clinical translation of experimental findings into humans. These innovative and noninvasive approaches have the advantage of monitoring the dynamic changes of neuroinflammation in epilepsy. Here, we will review the available evidence for the measurement of neuroinflammation in patients with epilepsy using noninvasive techniques and critically analyze the major scientific challenges of noninvasive methods. Finally, we propose the potential for use in clinical applications.

## 1. Introduction

Epilepsy is a common heterogeneous disease with a complex pathophysiology. Increasing evidence suggests that dynamic changes of neuroinflammation processes in epilepsy with a range of etiologies lead to the development and progression of this disease. Activation of microglia and astroglia triggers the release of inflammatory mediators including cytokines and chemokines. Initiation of inflammatory pathways exacerbates blood-brain barrier damage (BBBD) and fuels the innate and adaptive immune response within the brain and the periphery. These inflammatory processes often occur and last throughout the development of epilepsy, which contribute to the progression and severity of epilepsy. Recurrent epilepsy can also exacerbate brain inflammation. The causal and reciprocal link between neuroinflammation and epilepsy may contribute to neuronal hyperexcitability and drug resistance [1].

Modulation of these inflammation mechanisms could be a potential therapeutic target for epilepsy, which fostered interest in developing drugs targeting pathologic inflammatory pathways for selected epilepsy syndromes [2]. Identification of biomarkers of pathological neuroinflammation could help to define the patient population that is likely to benefit and the best treatment time for specific anti-inflammatory drugs [3]. Thus, there is an urgent need to develop clinically useful biomarkers that can predict the progression of neuroinflammation in patients with epilepsy and treatment response. How to measure and quantify brain inflammation in humans? The neuropathological observations of brain tissue from epilepsy surgery are the gold standard, but these samples are not routinely available. The biomarkers of cerebrospinal fluid (CSF) represent neuroinflammatory, but CSF obtained by lumbar puncture is invasive. Importantly, patients often reject invasive examination. Therefore, research has focused on the search for noninvasive biomarkers of neuroinflammation in various neurological disorders, including epilepsy [4].

Inflammatory mediator measurement in the blood sample and brain imaging of neuroinflammation could provide noninvasive methodologies to detect and quantify brain inflammation in humans. Blood samples and molecular neuroimaging are accessible and can be monitored repeatedly. Preclinical and clinical studies have developed potential biomarkers of neuroinflammation in epilepsy [3]. In this article, we will review the existing evidence measuring neuroinflammation with noninvasive techniques in epilepsy and critically analyze the major scientific challenges of noninvasive methodologies. Finally, we will address the suggestion that multidimensional biomarker panels can be used to identify brain inflammation in humans.

## 2. Blood Biomarkers

Immune cell subset distribution and inflammatory molecules in peripheral blood are candidate biomarkers. These biomarkers can be quantitatively measured and be used to evaluating brain inflammation progression or reaction to intervention. Mounting evidence has been made in identifying circulating neuroinflammatory biomarkers in animal models of epilepsy [5]. However, a major scientific challenge is to define valid and useful biomarkers in human epilepsy with efforts to ensure that individuals can benefit from immunomodulatory therapies.

### 2.1. Immune Cell Subset Distribution in Peripheral Blood

Changes in the immune cell subtypes indicate the activation of the immune system [6]. BBBD mediates the reciprocal brain-to-blood communication. Experimental studies of status epilepticus have demonstrated a pathogenic role of infiltrating monocytes [7]. Previous studies found infiltration of monocytes and lymphocytes in human brain tissue from epilepsy surgery with various etiologies [8–11]. In resected brain tissues from pediatric epilepsy patients, Xu et al. observed significant brain infiltration of peripherally derived T lymphocytes [12]. A recent work has shown that monocyte infiltration can contribute to the recurrence of epileptic seizures [13]. As the availability of brain specimens in epilepsy surgery is limited, blood provides the most easily accessible specimens for detecting the role of the immune system.

Flow cytometry remains a relatively popular method to investigate monocyte populations. Several cohorts reported differences in the profile of peripheral immune cells in epilepsy patients by cell sorting measurements of leukocytes [14, 15]. Decreased CD4^+^ T cells and increased NK cells were pronounced postictally in mesial temporal lobe epilepsy with hippocampal sclerosis [14]. Some studies showed an activation of classical monocytes [16] or an increase of the frequency of all monocytes [15]. A recent finding showed that the blood CD4^+^/CD8^+^ T cell ratio was elevated in patients with epilepsy due to limbic encephalitis compared to temporal lobe epilepsy (TLE) patients [17]. Compared with the control group, patients with TLE revealed distinct shifts in monocyte and lymphocyte subsets in the peripheral blood and CSF by flow cytometry. Changes in blood immune signatures were the most robust parameters that differentiated TLE from controls [18], including a shift toward immature CD14^low^CD16^+^ cells within monocytes, increased proportions of granulocytes, and decreased CD8^+^ T lymphocytes, while there was a weak negative correlation between CSF leukocyte count and time since the last seizure. Differently, the correlation of immune signatures with disease duration was not found. The clinical evidence supports that immune cell signatures may persist shift and the immune signature of TLE appears to manifest early in the disease course.

As studies on immune cells in the peripheral blood in patients with epilepsy syndrome are lacking, little is known about monocyte function in epileptogenesis. More information is still needed to understand whether these changes could be used as meaningful and reliable biomarkers of neuroinflammatory traits in epileptic syndromes [5].

### 2.2. Cytokine Levels in Peripheral Blood

Evidences from experimental and clinical research have supported that neuroinflammation is a hallmark of the epileptic focus in refractory epilepsy [5]. Cytokines are critical in immune regulation. Activation of cytokines and multiple pathways plays important roles in the development of chronic neuroinflammation during epilepsy [19]. Recent studies have shown a crucial contribution of glial cells (astrocyte and microglia) in the production of proinflammatory cytokines. The most commonly studied IL-1*β*, IL-6, and TNF-*α* tend to be potential mediators in the neuropathology of epilepsy [20]. Thus, considerable effort has been invested in the noninvasive identification of these neuroinflammation biomarkers.

It is interesting to note that the expression level of inflammatory cytokines varies with the cause and period of epilepsy. For example, serum proinflammatory cytokines increased after repetitive seizures, especially in cases of new-onset refractory status epilepticus or febrile infection-related epilepsy syndrome. Serum levels of IL-6 and TNF-*α* were detected with increased expression within 48 h in pediatric patients with acute afebrile seizures. The increased expression of cytokine levels (IFN-*γ*, IL-1*β*, and IL-6) in acute seizures was associated with younger patients at disease onset. The result suggested that younger patients showed stronger inflammatory responses to seizures. Correlation analysis showed that serum levels of IL-1*β* were significantly associated with disease severity in children with epilepsy. This set of evidence highlights that serum IL-1*β* may represent a biomarker for epilepsy as an ongoing neuroinflammation [21]. An observational study [22] reported that IL-6 levels in both serum and CSF were elevated in refractory status epilepticus and acute seizures. IL-6 levels normalized after tocilizumab treatment and clinical symptoms improved [23]. This phenomenon supports that IL-6 is a potential useful biomarker of inflammation and a measure of therapeutic response in this clinical entity.

An in vitro study suggested that after epilepsy, IL-1*β* mRNA, IL-6 mRNA, and TNF-*α* mRNA were expressed by microglia and astrocyte. The expression of IL-1*β* increases epilepsy susceptibility and neuronal excitability by directly inhibiting GABA_A_ receptor and promoting the phosphorylation of NR2B subunit of NMDA receptor. Low concentrations of IL-1*β* may exert antiepileptic effects by limiting intracellular Ca^2+^ and enhancing GABAergic transmission. The complex of IL-6 and IL-6 receptor can trigger gp130 signaling, which may disrupt cholinergic and GABAergic transmission of hippocampal neurons. Lowering extracellular Ca^2+^ levels can block the overexpression of IL-6. TNF-*α* can activate two receptors (p55 and p75). Low concentrations of TNF-*α* trigger apoptosis signal-regulating kinase 1 through the p55 pathway and induce neuronal apoptosis following seizures. High concentrations of TNF-*α* can play an antiepileptic role through the p75 pathway that associated with activation of the nuclear factor Kappa B (NF-*κ*B) system [20, 24]. However, these results are based on animal studies while cytokines in human epilepsy remain to be studied because cytokines can only be detected in blood or CSF. Further questions to be addressed are the extent to which cytokines are associated with human epilepsy and whether these pathways can be blocked by immunomodulatory therapy.

As the structurally related members of the immunoglobulin supergene family, intercellular adhesion molecules (ICAMs) organize a variety of junctions between cells and extracellular matrix, which mediate the cell signaling cascades on inflammation [25, 26]. Of the five ICAMs identified, soluble intercellular adhesion molecule 1 (sICAM-1) is the most widely studied inflammatory mediator and is activated in epileptic patients. Compared with drug-responsive epilepsy, serum sICAM-1 level was elevated in drug-refractory epilepsy. sICAM-5 is a kind of neuron-specific anti-inflammatory protein that plays an important immunosuppressive role in neuronal inflammatory diseases [27]. sICAM-5 can also be found in the blood that it can be a biomarker to detect the inflammatory response of epilepsy. Blood concentrations of sICAM-5 are reduced in epilepsy patients. T thymus and activation-regulated chemokine (TARC) levels have a growing trend in epilepsy. The ratio of TARC to sICAM-5 provides candidate blood biomarkers for refractory epilepsy and can be used for distinguishing epilepsy from normal controls [28].

Another cell adhesion molecule in the immunoglobulin superfamily, vascular cell adhesion molecule (VCAM), is a marker mainly expressed on the surface of endothelial cells that majorly regulate leukocyte adhesion and transendothelial migration, which mediates the process of vascular inflammation [29]. Soluble vascular adhesion molecules (sVCAM) mirror parenchymal inflammation in epilepsy. Clinical studies have demonstrated the upregulation of sVCAM in the serum and CSF of patients with epilepsy. CSF sVCAM-1 and serum sVCAM-1 levels were higher in the epilepsy group than in the neurosis group [30]. Moreover, there are higher CSF sVCAM-1 and serum sVCAM-1 concentrations in drug-refractory epilepsy compared to drug-responsive epilepsy. CSF and serum sVCAM-1 implied the possibility of drug resistance epilepsy and might be prognostic biomarkers for epilepsy.

Promising developments have been made in blood cytokines as biomarkers reflecting neuroinflammation in epilepsy, but caution should be taken. There are several drawbacks in these types of measurements. First, it is difficult to demonstrate that blood biomarkers meaningfully represent the degree and extent of brain inflammation. Second, seizures affect serum levels of cytokines, which may show seizure-dependent increase or decrease [31]. Third, since the half-life of many inflammatory cytokines is rapid, the blood levels vary considered and it is difficult to be accurately detected. CSF measurements of the inflammatory molecules would directly reflect brain inflammation released from the epileptic zone. However, these samples are not routinely available. Therefore, analysis of serum extracellular vesicles (EVs) derived from neuron and glia cells has received considerable attention as they can be measured through a noninvasive approach [32].

### 2.3. Serum Inflammatory Exosomes

Brain-derived EVs cross the BBB and can also be found in the peripheral blood [32]. Neuron-, astrocyte-, and microglia-derived EVs (NDEVs, ADEVs, and MDEVs) are enriched with several disease-specific proteins and/or microribonucleic acids (miRNAs). Therefore, serum EVs are a set of valuable biomarkers which noninvasively detect brain function and the progression of brain diseases [33]. Such a liquid biopsy approach makes it easier to repeat measures in clinical trials, convenient for testing the molecular mechanisms of the disease, the progression of the disease, and efficacy of treatment.

There have been only a few studies on the analysis of blood EVs in epilepsy [34, 35]. Yan and colleagues examined plasma miRNA-derived EVs in 40 patients with mesial temporal lobe epilepsy with hippocampal sclerosis (mTLE-HS) and 40 normal controls [36]. Expressions of over 50 EV miRNAs were abnormal in the plasma of these patients compared with healthy controls. In EVs from patients with mTLE-HS, miR-3613-5p and miR-6511b increased as much as 11-fold and 2-fold, respectively. Other 48 miRNAs showed downregulation. Five candidate EV miRNAs significantly decreased, including miR-4668-5p, miR-8071, miR-197-5p, miR-4322, and miR-6781-5p. Evidence indicated that they were involved in seizure development in mTLE-HS. Among these miRNAs, plasma EV miR-8071 differentiated mTLE-HS from healthy controls with a sensitivity of 83.3% and a specificity of 96.7%. In addition, miR-8071 was well associated with seizure severity. Therefore, plasma EV miR-8071 could represent a key diagnostic and prognostic marker for TLE-HS. Other clinical reports [35] have shown plasma miR-27a-3p, miR-328-3p, and miR-654-3p in exosomes as diagnostic markers with favorable sensitivity and specificity in patients with temporal lobe epilepsy. Specifically, the targets of the three miRNAs were associated with signaling pathways of neuronal apoptosis and growth factors involved in inflammation.

Notably, subtype analysis of astrocyte-derived exosomes in the serum has received considerable attention for evaluating brain inflammation [37]. Upregulation of inflammatory A1-type astrocyte exosomes, glial fibrillary acidic protein- (GFAP-) positive, plays an essential role in human inflammatory and neurodegenerative diseases of the CNS [38]. New findings support that A1-type astrocytes secrete neuronal toxic mediators which are pathogenically critical in human neurodegenerative diseases. Multiple studies have demonstrated that activated inflammatory A1-type astrocytes generate proinflammatory cytokines in the epileptic hippocampus [39–41]. However, little has been done to examine the A1 and A2 subtypes of astrocyte-derived exosomes in patients with epilepsy. The subtype studies of astrocyte-derived exosomes in the blood of patients with epilepsy could further help in evaluating the occurrence or progression of neuroinflammation and monitoring the effects of anti-inflammatory treatment. More studies are required on the role of exosomes in the pathophysiology of epilepsy.

### 2.4. Inflammasome Complex

As growing body of evidence suggests that complex signaling pathways are involved in neuronal excitotoxicity and cell loss progress during epilepsy, such as transforming growth factor- (TGF-) *β*, interleukin- (IL-) 1 receptor/Toll-like receptor (TLR), and cyclooxygenase-2 (COX-2) signaling pathways. Major research in recent years focuses on the expression of inflammasome complex and the influence on induced seizures in animal models of epilepsy, as well as findings in human studies [42]. Inflammasome is a multiprotein complex that has been understudied as a new target to neuroinflammation in epilepsy. It is mainly composed of NOD-like receptor protein (NLRP), apoptosis speck-like protein (ASC), and caspase 1 (CASP1), which are considered key platforms of inflammatory signaling pathway [42]. The NLRP3 inflammasome components, the most widely studied one, is mainly activated and expressed in the microglia and astrocytes after oxidative stress, hypoxia, or acidosis [43]. CASP1 can be activated by the interaction between NLRP3 and ASC, resulting in production of inflammatory cytokines such as IL-1*β*, IL-18, and TNF-*α*, which trigger a cascade of inflammatory response [24, 44]. The NLRP3/ASC/caspase 1 inflammation pathway leads to epileptic neuronal apoptosis, thereby promoting epileptogenesis, and ultimately developed into seizures and recurrence. In contrast to NLRP3, the NLRP1 mainly expressed in neuron. The activation of NLRP1 inflammasome component generates caspase 1 and leads to programmed cell death termed “pyroptotic death” [45]. Clinical studies have shown that in patients with TLE, NLRP3 and NLRP1 inflammasomes are upregulated and they are associated with the increased hippocampal expression of caspase 1 and IL-1*β*. Pharmacological inhibition of NLRP1, NLRP3, or caspase 1 can reduce seizure frequency and severity in TLE rats [46–48]. Components of the inflammasome pathway might be useful as biomarkers in neuroinflammation epilepsy and new targets of antiepileptogenic strategies in TLE patient while the transformation from animal studies to clinical trials needs further exploration considering that the drug treatment of human epilepsy is more complicated than animal models [44].

Overall, these studies are promising and imply that clinical translations of such noninvasive blood approaches are attractive for periodic analyses in different phases and types of epilepsy. However, several limitations remain. For example, lacking critical spatial information of the brain inflammation, indirectly reflecting the brain phenomenon, and the variability of peripheral blood reports are still considerable. Therefore, the combination of multiple blood biomarkers and brain imaging markers may enhance the diagnostic potential of neuroinflammation in epilepsy.

## 3. Brain Imaging Markers

### 3.1. TSPO PET

Translocator protein 18 kDa (TSPO), the peripheral benzodiazepine receptor on the outer mitochondrial membrane of microglia and reactive astrocytes [49], is upregulated by activated microglia [50] and reactive astrocytes, which is a promising biomarker of neuroinflammation [51]. TSPO positron emission tomography (PET) is the most widely studied noninvasive imaging to better characterize the neuroinflammatory processes underlying epilepsy [49, 52, 53].

TSPO has been shown to be upregulated in patients with TLE, neocortical epilepsy, and drug-resistant epilepsy, as well as in animal models [54–56]. Alterations in its expression indicate a different state of epilepsy. TSPO expression increases peak in the subacute phase (1-2 weeks) after the onset of epilepsy and maintains a certain concentration level in the chronic phase [57], which suggests microglia-mediated inflammation is involved in the occurrence and persistence of epilepsy, which could be further investigated by PET imaging [50, 52, 58]. For example, the study of patients with neocortical frontal epilepsy using the ^11^C-PK11195 TSPO PET tracer showed that inflammatory responses in brain lasted approximately 36 hours after seizure and the inflammatory areas were colocalized with the frontal epileptogenic zone [58]. Using ^11^C-PBR28 tracer, a study revealed that increased brain uptake of the tracer was evident in the ipsilateral hippocampus to the seizure focus than contralateral in TLE patients, including patients with mesial temporal sclerosis (MTS) [55]. In a rat model of status epilepticus (SE), TSPO PET using ^18^F-DPA-714 tracer showed increased uptake within the limbic system even in the hippocampus and reached its maximum at 7 days after SE, while TSPO binding declined to the baseline levels at 14-16 weeks post-SE. It demonstrated that TSPO binding changed over time in epilepsy with neuroinflammation [59].

To be more precise, TSPO PET could in vivo quantify the spatial temporal profile of microglial activation in patients with epilepsy and SE-induced rat models [60], which has the potential for determine the therapeutic windows in epilepsy and monitoring the response to anti-inflammatory treatment [58]. In rat models, early TSPO upregulation is associated with epileptogenesis, while chronic TSPO overexpression is related to seizure frequency [61]. TSPO PET can be used to ascertain spontaneous recurrent seizure frequency and reflect the severity of related comorbidities such as depression-like and sensorimotor-related disorders [52]. Meanwhile, TSPO PET also serves as an auspicious tool for temporal monitoring and quantification of anti-inflammatory effects of different drugs during epileptogenesis [62].

These findings further support the idea that TSPO PET might also be a valid biomarker for assessing epileptogenesis-associated brain inflammatory processes, and it would be particularly valuable that other imaging modalities are unrevealing [54–56]. However, there are still certain limitations to measure reliably neuroinflammation by PET imaging. PET tracer is one of the most important factors that affect the sensitivity of TSPO PET. The first-generated tracer ^11^C-PK11195 has several disadvantages such as limited brain entrance, poor signal-to-noise ratio, and labeling with the impractically rapidly decaying isotope that affects the specificity of TSPO detection [63]. Novel radiotracers have improved the ability to measure TSPO in vivo [64]. The second-generated tracers, such as ^18^F-DPA-714, ^11^C-PBR28, and ^18^F-PBR111, with better enhanced pharmacological and pharmacokinetic properties, offer more appropriate tools for in vivo TSPO-PET imaging [52]. In recent years, ^18^F-GE-180, the third-generated TSPO PET tracer, has been rapidly translated into human clinical research due to the advantages of higher signal-to-noise ratio and lower nonspecific binding. However, the current dispute refutes this view. The insensitive genotype seems to be blamed on poor quality of images, and higher signal-to-noise ratio is only because of the broken BBB. Thus, ^18^F-GE-180 is considered to have low credibility, even if it failed for TSPO protein detection [65].

Besides, TSPO signal in the brain varies between the normal intrasubject and a true reference region which is absent; it is difficult to accurately calculate the sample size for an anti-neuroinflammatory treatment study [58]. Increased TSPO expression signals may also be observed in nonepileptic lesions due to BBBD or due to more radiotracer availability in the blood, which may reduce the specificity [55]. Interestingly, TSPO was identified in both proinflammatory and anti-inflammatory tissues. Besides, TSPO binding should not be assumed to reflect specific microglial activation, as it is also expressed by astrocyte and vascular endothelium [62]. Future research should pay more attention to further screening novel PET radiotracers that will provide fascinating insights into the ability to measure TSPO in vivo and improve understanding of the meaning of the TSPO-PET results.

### 3.2. Gadolinium- (Gd-) Enhanced MRI

Besides microglia and astrocytes, BBBD, as well as named BBB leakage, is also tightly coupled to neuroinflammation [66]. In the experimental epilepsy model of animals, BBBD can promote epileptogenesis [3, 67]. Neuroinflammation may originate directly from the central nervous system or from the peripheral circulation due to the destruction of the BBB [68]. The leakage of plasma constituents to the extracellular neuronal environment leads to progression of neuroinflammation and enhanced cortical excitability [66, 67]. Noninvasive quantitative measures of BBBD are clinically required to reach a more accurate identification of neuroinflammation [69].

Increased vascular permeability (“leakiness”) of the disrupted BBB can be measured using gadolinium- (Gd-) enhanced MRI [63]. Under normal circumstances, gadolinium-based contrast agents do not cross the intact BBB. However, it may extravasate from the blood into the brain tissue even when BBBD occurs [70]. Thus, the contrast agents leaked from the circulation can be detected and quantified with high spatial resolution [71]. Breuer et al. [72] reported that the BBB leakage was detected by gadolinium- (Gd-) enhanced MRI at 1 day and 6 weeks after SE. BBB leakage is measured with Gd-enhanced MRI during early epileptogenesis, which can be a potential biomarker of later emerging epileptic seizures. During the chronic phase, BBBD has received increasing attention because of evidence of its association with an increased risk of seizure frequency. Therefore, BBBD may be used as a biomarker to monitor the efficacy of a potential therapeutic epilepsy treatment [73]. There is recent progress in the analysis of brain dynamic contrast-enhanced magnetic resonance imaging (DCE-MRI), in which the linear behavior of the contrast agents in the brain vasculature and parenchyma is used to evaluate BBB permeability [67, 74]. It showed higher values of DCE-MRI index in predicting lesions with a higher propensity to cause seizure recurrence [75].

For future studies, gadolinium- (Gd-) labeled contrast-enhanced MRI seems to be the most favorable modality to image BBB leakage with epilepsy [71, 72], However, most of the research on Gd-enhanced MRI stays in animal models because of the duration and frequency of seizures, as well as patient characteristics (age, medication, and concomitant conditions) may affect BBB permeability [72]. Besides, Gd-enhanced MRI measurements in clinical use are currently limited to measuring paracellular leakage of low molecular weight gadolinium contrast agents. Due to the low amplitude of signal change detected using these methods, some factors can confound the results of measurements, such as partial volume errors, Gibbs ringing, signal drift, patient motion, arterial input function definition errors, and kinetic model inaccuracy [76]. Of note, gadolinium- (Gd-) labeled contrast-enhanced MRI is characterized by potential toxicity. A large number of clinical and animal experiments have shown that multiple exposures to gadolinium-based contrast agent have health effects such as nephrotoxicity [77]. Thus, the current thinking regarding the permeability of the BBB may be greatly oversimplified and limited to animal models [70]. Additional investigations in the future are needed to clarify the relationship among different factors for neuroinflammation due to BBBD.

### 3.3. Magnetic Resonance Spectroscopy (MRS)

MRS can assess the neurochemical changes in given brain regions of interest and provide metabolic or inflammatory information of neurons and neuroglial cells in vivo without invasive intervention [78]. Proton MRS (^1^H-MRS) is one of the most common methods for MRS, and it can detect and quantify endogenous metabolites including N-acetyl aspartate (NAA, a marker for neuronal status and integrity), choline (Cho, a marker for membrane integrity and turnover), creatine (Cr, a marker for energy metabolism), myo-inositol (Ins, a marker for glial cell integrity), and glutamate^+^ glutamine (Glx, related to excitatory neurotransmission) [79]. ^1^H-MRS can be used to measure neuroinflammation, and its molecular biochemical detection principle can be used to assist to detect neuroinflammation in epileptic patients [63].

MRS could in vivo monitor the inflammation of epileptogenic foci in patients with epilepsy. A study has demonstrated significant reductions in the NAA/Cr and NAA/(Cr^+^Cho) ratios in the hippocampus ipsilateral to the epileptic zone in structured MRI-negative TLE patients [80]. The pathological outcome of the resected hippocampus suggested neuroinflammation. Magnetic resonance spectroscopy and thermometry (MRS-t) is a temperature imaging which is currently under study, and this technique can be used to monitor the inflammatory response of epileptic lesions. At the same time of neuroinflammation, the metabolic demand of brain tissue increases correspondingly, which may inhibit the cooling mechanism of brain and make the temperature of brain tissue 1-2°C higher than the core temperature. Therefore, MRS-t can be used to monitor the neuroinflammation of epilepsy and its response to treatment [63, 80].

However, the practicability of MRS in detecting epileptogenic inflammation is mainly limited by the intensity and power of the magnetic field, which affects the accurate quantification of different neurotransmitters [81]. It has been reported that ^1^H-MRS is applied to detect epilepsy ranging from TLE [82] to idiopathic generalized epilepsy while it seems to be of little value for monitoring insular epilepsy [83]. In addition, antiepileptic drugs also have a confounding effect on nerve metabolism and affect the monitoring effect of MRS [84]. To date, there are a few studies on detecting the dynamic changes of neuroinflammation by MRS in epilepsy and it has very limited resolution for the practical technical support [83, 85, 86].

## 4. Conclusion

A graphical abstract showing the main conclusions of this review is shown in Figure 1. The discovery of noninvasive biomarkers of maladaptive neuroinflammation in epilepsy would facilitate clinical translation of anti-inflammatory treatments as they would enable the identification of patients who could benefit from the treatments and would provide pharmacodynamic markers of the therapeutic response. Despite the present evidence of seizure reduction by anti-inflammatory drugs in humans that relies mostly on case reports or small series, the association between the disease and biological markers of altered immunity has been still found in these cases. Numerous questions need to be answered. This effort might provide powerful tools for epileptologists to make complex decisions regarding the anti-inflammatory treatment of selected epilepsy patients

Brain inflammation in epilepsy is based on multidimensional systems combining phenotypic, molecular variables, neuroimaging, and neuropathology. Since various biomarkers from blood and neuroimaging may carry complementary information, the fusion of multidimensional and multimodal biomarker features may be a promising option to improve the identification accuracy of brain inflammation in humans. The complex assessment of multidimensional biomarker panels will provide a wealth of information and guide decision-making in patients with epilepsy.

## Figures and Tables

**Figure 1:** Graphical abstract showing the main blood biomarkers and brain imaging markers suggesting neuroinflammation in epilepsy. IL: interleukin; TNF-*α*: tumor necrosis factor-*α*; ICAM: intercellular cell adhesion molecule; VCAM: vascular cell adhesion molecule; NLRP: NOD-like receptor protein; ASC: apoptosis speck-like protein; TSPO PET: translocator protein positron emission computed tomography; MRI: magnetic resonance imaging.

## Abbreviations

CSF: Cerebrospinal fluid
BBBD: Blood brain barrier dysfunction
TLE: Temporal lobe epilepsy
ICAMs: Intercellular adhesion molecules
sICAM-1: Soluble intercellular adhesion molecule-1
TARC: T thymus and activation-regulated chemokine
VCAM: Vascular cell adhesion molecule
EVs: Extracellular vesicles
miRNAs: Microribonucleic acids
mTLE-HS: Mesial temporal lobe epilepsy with hippocampal sclerosis
NLRP: NOD-like receptor protein
ASC: Apoptosis speck-like protein
CASP1: Caspase 1
TSPO: Translocator protein
PET: Positron emission tomography
MTS: Mesial temporal sclerosis
SE: Status epilepticus
DCE-MRI: Dynamic contrast-enhanced magnetic resonance imaging
MRS: Magnetic resonance spectroscopy.
